# Outcomes of Visualized Puncture Needle and Small Needle-Knife Therapy in Primary Frozen Shoulder Based on Multimodal Ultrasound Imaging

**DOI:** 10.1155/2022/1076112

**Published:** 2022-02-16

**Authors:** Xin Qin, Baoli Zhang, Yan Feng, Xiaoping Gao, Zhihong Liu, Yanxia Yang, Qiang Liu

**Affiliations:** ^1^Northwest Minzu University, No.1 Xibei New Village, Chengguan District, Lanzhou City, Gansu Province 730030, China; ^2^Gansu University of Traditional Chinese Medicine, Lanzhou, Gansu 730000, China

## Abstract

**Objective:**

To compare the outcomes of visualized puncture needle and small needle-knife therapy in 68 patients with primary frozen shoulder.

**Method:**

Sixty-eight patients with primary frozen shoulder were recruited and randomly divided into two groups, with 34 patients in each group. In the treatment group, an ultrasound-guided 18G-PTC puncture needle was inserted into the joint space, followed by a liquid injection until complete lysis and dissociation of the intraarticular adhesion were achieved. Then, the lesser tuberosity of the coracoid and humerus, the intertubercular groove of the humerus, and the greater tuberosity of the humerus were stripped, first vertically and then horizontally, by an amplitude ≦ 0.5 cm per treatment. This treatment procedure was performed once per week, and each cycle covered three treatments. The small needle-knife therapy was set as a control, and the efficacy was observed.

**Result:**

The visualized puncture needle significantly outperformed the small needle-knife therapy in overall efficacy, UCLA scores of the shoulder joint, shoulder mobility, and muscle elasticity and thickness.

**Conclusion:**

The efficacy of the visualized puncture needle for primary frozen shoulder was better compared to the small needle-knife therapy. The former was safer and more convenient, which caused less pain to patients and took effect more quickly. In a word, the visualized puncture needle for primary frozen shoulder is worthy of clinical popularization.

## 1. Introduction

Primary frozen shoulder is also known as idiopathic periarthritis of the shoulder, and its etiology is not yet fully clarified. This disorder mainly presents with restricted mobility of the shoulder joint, osteoporosis of the glenohumeral joint, and ossifying myotenositis [1]. Many patients seek medical care due to unbearable pain and restricted mobility of the shoulder joint. Primary frozen shoulder is a common disease in clinical practice. The chronic intracapsular inflammation of the shoulder joint leads to continuous infiltration of the lower layer of the synovium, resulting in fibrosis and intracapsular adhesion. Consequently, the mobility of the joint is lost. Besides, the inflammation may be further aggravated as fibrosis progresses, promoting abnormal proliferation of the nerve cells and leading to pain sensitivity. The abovementioned changes hinder patient rehabilitation, triggering the vicious cycle of pain, immobility, adhesion, and pain aggravation. At present, the treatments for primary frozen shoulder cover surgical and conservative treatments. Conservative treatments mainly include medication, acupuncture, massage, and physical therapy, which aim to relieve pain and restore joint mobility. Surgical treatment mainly refers to the removal of the adhesion. However, both have shortcomings. Small needle-knife therapy is less invasive, fast acting, and convenient, which has been widely applied to periarthritis of the shoulder as it shortens the treatment time and reduces treatment frequency and patients' pain. However, there have been reports of disease aggravation due to accidental injury of blood vessels and nerves. Thus, there are risks for small needle-knife therapy. We reviewed the literature comprehensively, and the visualized puncture needle was selected as an alternative for the small needle-knife therapy. The surgery using the visualized puncture needle was performed under ultrasound guidance to avoid injury of the blood vessels and nerves, and satisfactory outcomes were demonstrated by the multi-modal ultrasound imaging.

## 2. Clinical Data

### 2.1. General Information

Sixty-eight patients with primary frozen shoulder treated at our hospital from March 1 to November 30, 2020, were recruited. The protocol was approved by the ethics committee. The patients were divided into two groups using a random number table, with 34 patients in each group. From inquiry and measurement, the detailed information is as follows: There were 21 males and 13 females in the treatment group. The eldest was aged 72 years old, and the youngest was 43 years old, with an average of 53.34 ± 7.83 years. The longest course of disease was 32 weeks, and the shortest course was 8 weeks, with an average of 16.27 ± 7.13 weeks. As to the side affected, 28 patients were affected unilaterally and 6 patients bilaterally. There were 19 males and 1 female in the control group. The eldest was aged 70 years old, and the youngest was 44 years old, with an average of 54.61 ± 7.58 years. The longest course of disease was 33 weeks, and the shortest course was 8 weeks, with an average of 16.27 ± 7.13 weeks. As to the side affected, 21 patients were affected unilaterally and 13 patients bilaterally. There were no significant differences in baseline parameters between the two groups (*P* > 0.05).

### 2.2. Diagnostic Criteria

#### 2.2.1. Diagnostic Criteria of Western Medicine

The diagnostic criteria developed by Shin SJ [2] were used, which are as follows: (1) pain around the shoulder with restricted mobility for ≥4 weeks; (2) shoulder joint pain interfering with daily living or work; (3) night pain; (4) restricted mobility of the shoulder joint, particularly restricted active or passive raising or external rotation; (5) no abnormal radiological findings; and (6) no secondary factors.

#### 2.2.2. Diagnostic Criteria of Traditional Chinese Medicine

The Criteria for Diagnosis and Treatment of Syndrome of Internal Medicine of Traditional Chinese Medicine (National Administration of Traditional Chinese Medicine, 2012 edition) were used for the diagnosis in the present study, which are as follows [3]: (1) chronic strain or bone injuries, with the wind-cold damp pathogen invading before qi and blood recovery; (2) the vulnerable age group is 50–60 years, and the disease is more common in females than in males, especially among the manual workers. The patients usually have a chronic onset; (3) pain around the shoulder joint, especially at night. The pain is usually induced by changes in weather and fatigue, resulting in shoulder joint dysfunction; (4) shoulder muscle atrophy, with tenderness in the shoulder front, back, and lateral sides. The abduction is restricted significantly, presenting with a typical abducting-shoulder lifting phenomenon; (5) X-ray findings are usually negative, and those with a longer course of disease are usually combined with osteoporosis.

### 2.3. Inclusion Criteria

The inclusion criteria were as follows: (1) meeting the western and traditional Chinese medicine criteria for primary frozen shoulder; (2) explicit history of primary frozen shoulder; (3) persistent shoulder pain for over 4 weeks; (4) tolerant to small needle-knife therapy and visualized puncture needle; and (5) cooperative with the study and completing all the scheduled procedures to ensure that the study data were intact and reliable.

### 2.4. Exclusion Criteria

The exclusion criteria were as follows: (1) restricted mobility or pain of the shoulder joint due to shoulder deformity, fracture, ligament damage, surgery or trauma; (2) bone and joint diseases of the neck; (3) severe dysfunction of other major organs; (5) skin damage of the shoulder; (6) history of allergy or allergic to the test drug; and (7) poor compliance to the treatment or lost to follow-up.

### 2.5. Elimination Criteria

The elimination criteria were as follows: (1) severe adverse events during clinical observation, which threatened patients' recovery or life; (2) the development of other disorders or complications during clinical observation, which affected the results; (3) poor compliance and failure to complete the scheduled procedures; (4) quitting the treatment for other reasons; and (5) receiving other treatments during the study, which affected the results (e.g., receiving other medication or other treatments). Patients meeting any of the abovementioned criteria were eliminated.

### 2.6. Dropout Criteria

Dropouts were defined as patients who withdrew from the study or were lost to follow-up. The dropouts were eliminated from the analysis.

### 2.7. Treatment Procedures

In the puncture group the patients took a prostrate position. The skin around the shoulder joint was disinfected routinely. The probe was wrapped in a sterile probe (Philips iU22 ultrasound system, with a high-frequency probe at 5–12 MHz), which was placed horizontally behind the shoulder joint to trace the incisure of the humeral head, posterior labrum, and spinoglenoid. An 18 G/21G-PTC puncture needle (connected with a 20 ml syringe, filled with 5 mg of triamcinolone acetonide plus 15 ml of normal saline) was inserted into the joint space lateroposteriorly under ultrasound guidance. After confirming that there was no blood return, the liquid was slowly injected into the joint space from the syringe. It was observed by ultrasound whether the intraarticular adhesion was completely removed. Then, the needle was withdrawn, and the needle path was blocked. The lesser tuberosity of the coracoid and humerus, the intertubercular groove of the humerus, and the greater tuberosity of the humerus were stripped first vertically and then horizontally, under the ultrasound guidance by an amplitude of ≤0.5 cm per treatment. This was followed by an injection of 20 ml of triamcinolone acetonide (0.5 ml). The procedure was performed once per week, with each cycle covering three treatments.

In the small needle-knife therapy group, the patients took a sitting position, with their hands placed on the back of the chair. The lesser tuberosity of the coracoid and humerus, the intertubercular groove of the humerus, and the greater tuberosity of the humerus were located. Local anesthesia was performed using 1 ml of 0.2% lidocaine hydrochloride injection per point. The four-step small needle-knife therapy was conducted using the Huatuo 1.0∗80 mm disposable sterile medical needle-knife at the following sites: (1) Coracoid: the knife edge was aligned with the long axis of the humerus. The needle-knife was inserted to the vertex of the coracoid until it reached the bone surface. The stripping was performed vertically and then horizontally. (2) Lesser tuberosity of the humerus: the knife edge was perpendicular to the skin. The direction of insertion was aligned with the orientation of the subscapular muscle. The knife was directly inserted to the lesser tuberosity of the humerus to perform the stripping, first vertically and then horizontally. (3) Intertubercular groove of the humerus: the knife edge was aligned with the long axis of the humerus. The knife was directly inserted into the plane of the intertubercular groove of the humerus to perform the stripping, first vertically and then horizontally. (4) Greater tuberosity of the humerus: the line of the knife edge was aligned with the long axis of the humerus. The small needle-knife was inserted all the way to the bone below the greater tuberosity of the humerus for lifting-thrusting and lysis. The treatment was performed once per week, with each cycle covering three treatments.

### 2.8. Efficacy Indicators and Observation

#### 2.8.1. Overall Efficacy Observation

The overall efficacy for primary frozen shoulder was evaluated according to the Criteria for Diagnosis and Treatment of Syndrome of Internal Medicine of Traditional Chinese Medicine [3]. Cure: no local swelling or pain, with the normal joint function completely restored. Improved: mild local swelling or pain, with the joint function partially restored. Uncured: the symptoms or signs are not improved after treatment or even aggravated. Overall response rate = (number of patients cured + number of patients achieving an improvement)/total number of patients×100%.

#### 2.8.2. Shoulder Scores

The UCLA shoulder rating scale [4] was used, and the total score was 35, with 10 for function and 10 for pain. The total score was 5 for active forward flexion, active forward mobility, and patient satisfaction, respectively. Three categories were classified based on the total score: 34–35 indicated excellent, 29–33 fairly good, and <29 poor. The efficacy was compared between the two groups based on the UCLA scores. Note: excellent UCLA score, marked efficacy; fairly good score, efficacy; and poor score, inefficacy.

#### 2.8.3. Shoulder Mobility

Abduction, adduction, and extension of shoulder joints in the two groups were measured before, during, and after the treatment [5].

#### 2.8.4. Shoulder Joint Pain

The shoulder joint pain was assessed using the visual analog scale (VAS) [6].

#### 2.8.5. Muscle Elasticity and Thickness Determined by Ultrasound Elastography

At each time point, the iU22 ultrasound system was used for ultrasound elastography along with a high-frequency probe (4.0–9.0 MHz) and quasistatic ultrasound elastography software. Specifically, MSK sonography was performed three times by one ultrasound doctor for each patient, and an average was taken. The elasticity *E* value is a basic parameter reflecting muscle elasticity and hardness. The formula is as follows: *E* = *S*/*e*, where S is the external pressure applied; *e* is the degree of deformation upon compression. The larger the *E* value, the lower the tissue elasticity would be. The smaller the *E* value, the higher the tissue elasticity would be. To measure the muscle thickness, the patient took a sitting position and tried to be relaxed as much as possible. The linear array probe was positioned to measure the thickness of the supraspinatus muscle at its highest point at the 1/2 position of the line connecting the acromion and the root of the neck. The thickness of the infraspinous muscle was measured at the 1/2 position of the line connecting the mesoscapula and the inferior horn of the scapula [7].

### 2.9. Statistical Analysis

Statistical analyses were conducted using the SPSS 22.0 software. ANOVA was conducted. Measurements were compared using the *t*-test and counts *χ*^2^ test.

## 3. Results

### 3.1. Efficacy Observation

The overall response rate of the puncture needle group was 88.23% compared to 67.64% in the small needle-knife therapy group, with a significant difference (*P* < 0.05). The overall response rate of the ultrasound-guided puncture needle therapy group was higher than that of the small needle-knife therapy group (Table 1).

### 3.2. Shoulder Scores at Different Time Points

There were no significant differences in the shoulder scores between the two groups at the baseline (*P* > 0.05). The shoulder scores were improved significantly in the two groups after treatment (*P* < 0.05). Besides, the efficacy of the ultrasound-guided puncture needle therapy was considerably better compared to the small needle-knife therapy (*P* < 0.05) (Table 2).

### 3.3. Observation of Shoulder Mobility

Before the treatment, there were no significant differences in the range of motion of abduction, forward flexion, and backward extension between the two groups (*P* > 0.05). During treatment, the range of motion of abduction was improved in the puncture needle group after the first treatment (*P* < 0.05). Besides, as more treatments were provided, the joint mobility was further improved (*P* < 0.05). The efficacy of the puncture needle group was better compared to that of the small needle-knife therapy group (*P* < 0.05). The range of motion of forward flexion was improved in the puncture needle group after two weeks of treatment (*P* < 0.05), which was maintained at the end of treatment (*P* < 0.05). As to backward extension, there was a response in the puncture needle group only at the end of treatment (*P* < 0.05) (Table 3).

### 3.4. Pain Assessed by VAS

Before the treatment, there were no significant differences in the VAS scores between the two groups (*P* > 0.05). As more treatments were provided, the VAS scores decreased significantly in the puncture needle group (*P* < 0.05), indicating pain relief. Besides, the VAS scores were improved significantly in the puncture needle group than in the small needle-knife therapy group (*P* < 0.05). These results suggested that the visualized puncture needle therapy relieved the pain more effectively (Table 4).

### 3.5. Muscle Elasticity and Thickness Measured by Ultrasound Elastography

Before the treatment, the thickness of the supraspinatus and infraspinatus muscles was not significantly different between the two groups (*P* > 0.05). The puncture needle group achieved a response in the supraspinatus muscle thickness only after 2 weeks of treatment, with a significant difference (*P* < 0.05). The difference became even more prominent after 3 weeks of treatment. At this time point, although the average supraspinatus muscle thickness had changed in the small needle-knife therapy group, the difference was not statistically significant (*P* > 0.05). The changes in the infraspinatus muscle thickness were not obvious in either group during the treatment. The difference was only statistically different in the puncture needle group after 3 weeks of treatment (*P* < 0.05) (Table 5).

Before the treatment, the elasticity *E* values of the supraspinatus and infraspinatus muscles were not significantly different between the two groups (*P* > 0.05). The elasticity of the supraspinatus muscles was improved significantly in the puncture needle group after 2 weeks of treatment (*P* < 0.05). For the small needle-knife therapy group, the elasticity of the infraspinatus muscles was not significantly improved at the end of treatment (*P* > 0.05). The elasticity of the supraspinatus muscles was improved significantly in the puncture needle group only after 3 weeks of treatment (*P* < 0.05). Besides, the difference was statistically significant compared with the small needle-knife therapy group (*P* < 0.05) (Table 6).

## 4. Discussion

Primary frozen shoulder is a self-limited disease for which the pathogenesis remains unknown. This disease usually affects those aged around 50, and most patients do not have a history of trauma. Primary frozen shoulder initially presents with shoulder pain, followed by progressive restricted mobility. The patients may finally develop a frozen shoulder joint and cannot move or suffer from pain upon movement. This disorder is known as frozen shoulder or shoulder palsy, and falls into the category of arthralgia in traditional Chinese medicine. The primary pathogenesis of arthralgia includes stagnation of Qi and blood and blockage of vessels, resulting in pain. According to the syndrome differentiation in traditional Chinese medicine, the pathogenesis of frozen shoulder is attributed to the invasion of external evils (wind, cold, dampness, and heat) or the damage of the meridian-sinews, collaterals, and subcollaterals or even channels due to fatigue and internal injury. There is an insufficient promotion of channel Qi to nourish the shoulder joint, which further results in Qi and blood stagnation. As Qi and blood block the vessels, pain is elicited. Besides, the deficiency of Qi and blood also causes loss of nourishment in the meridian-sinews around the shoulder joint, leading to progressive contracture. The function of the shoulder joint is finally lost, which becomes frozen. According to the views of modern Western medicine, subacromial bursal tissue inflammation mediated by inflammatory factors [8] is an important pathological process associated with primary frozen shoulder. As the chronic inflammation develops, fibrotic hyperplasia occurs within the shoulder joint capsule [9], which affects the articular cavity and joint mobility. In the meantime, calcitonin gene-related peptide (CGRP) and substance P (SP) [10] in the shoulder joint capsule generate abnormal nerve fibers under the inflammatory immune response, which serves as the pathological basis for intracapsular pain. Shoulder joint pain further decreases joint pain and mobility. The patients may present with muscle atrophy around the shoulder, tendon fibrosis (calcification), and joint capsule atrophy, leading to a vicious cycle. As a result, most of the shoulder function is lost. In other words, the key pathogenesis associated with primary frozen shoulder is inflammation-induced joint fibrosis and the resulting adhesion. Therefore, the treatment of primary frozen shoulder is to remove the adhesion.

At present, the views of traditional Chinese medicine and Western medicine diverge dramatically regarding the treatment of the primary frozen shoulder. Western medicine recommends oral painkillers (including nonsteroidal anti-inflammatory drugs) for patients with mild or severe pain [11]. Surgery is recommended for severely affected patients [12] to remove joint adhesion, followed by rehabilitation exercise of the shoulder joint to promote functional recovery. Although surgery can temporarily remove shoulder adhesion, postoperative rehabilitation exercise is strenuous, painful, and takes time. Many patients fail to pursue rehabilitation exercises in the midway and then develop joint adhesion again. The disorder upon the secondary adhesion is usually more serious than before surgery. Postoperative infection may also lead to treatment failure. For these reasons, surgery is mainly indicated for patients with severe shoulder adhesion and complete loss of function. Traditional Chinese medicine recommends treatments addressing etiology and symptoms based on pathogenesis. The wind, cold, and dampness evils in the shoulder joint are removed and the channels are dredged by acupuncture [13], hot compress [14], and plaster. These procedures can promote Qi and blood circulation and facilitate the local movement of Qi as etiological treatments. Besides, the passive movement of the shoulder joint is promoted by massage and traction to restore normal shoulder mobility. This is a major strategy for conservative therapy, which is also the primary treatment for those with mild disease or a shorter course of disease. However, there are also the problems of long-term treatment, high risk of recurrence, and painfulness. Small needle-knife therapy was first put into clinical practice in the 1980s, which has already been recognized by clinicians due to its simplicity of operation, small invasiveness, less damage, and good efficacy. Hence, this procedure has been widely applied to a variety of meridian sinew diseases. Small needle-knife therapy is mainly indicated for primary frozen shoulder [15], and many related reports have been published. However, there are also risks for small needle-knife therapy, such as accidental injury of blood vessels and nerves, and unintended damage of normal and fibrous tissues and the articular surface, which directly affect the efficacy and even aggravate the disease.

Based on the clinical experience, the authors have found that the ultrasound-guided puncture needle can avoid the adjacent blood vessels and nerves and reach the lesion directly. In this way, the visualized puncture needle therapy can prevent risks otherwise associated with small needle-knife therapy while achieving the therapeutic goals. The former also allows for the local drug administration or extraction of articular cavity fluid, rendering it eligible to replace the small needle-knife therapy. Besides, through a literature review, we have found that many reports are related to the clinical application of puncture needle therapy. Based on existing literature and our own experience, we developed a modified puncture needle therapy and aimed to replace the needle-knife with the puncture needle. First, the puncture needle was used for intracapsular injection of triamcinolone acetonide and normal saline under ultrasound guidance to loosen the joint adhesion via hydraulic dilation. Next, a procedure similar to that used in small needle-knife therapy was performed to strip the lesser tuberosity of the coracoid and humerus, the intertubercular groove of the humerus, and the greater tuberosity of the humerus to relieve contraction of the peripheral meridian-sinews. This step was accompanied by a local administration of lidocaine for pain relief. The efficacy was then compared between the small needle-knife therapy group and the puncture needle group, and it was found that the efficacy of the puncture needle group was better (*P* < 0.05). Specifically, the puncture needle group improved the intracapsular adhesion, forward flexion, and abduction of the forelimbs more effectively. This result could be explained by the hydraulic dilation caused by the puncture needle inserted into the joint cavity to remove the adhesion. Moreover, muscle fibrosis was relieved by the procedure similar to that used in small needle-knife therapy at the important points around the shoulder. As indicated by the changes in local muscle elasticity and thickness, the muscle function was gradually restored as the shoulder mobility was improved. Accordingly, the muscle tone was increased in the atrophic muscle group of the shoulder and finally restored to normal. Besides, as the intracapsular adhesion was removed or mitigated, the secretion of intraarticular neurotransmitters such as SP and CGRP was decreased, and the growth of the immunopositive nerve fibers was decreased as well. Therefore, the shoulder pain was mitigated, and the VAS score was improved significantly. The UCLA shoulder scores indicated that the efficacy of the ultrasound-guided puncture needle was better than that of the small needle-knife therapy for primary frozen shoulder. Taken together, the efficacy of the visualized puncture needle therapy was better for primary frozen shoulder compared to the small needle-knife therapy. The former is safer and more convenient, which causes less pain to patients and takes effect quickly. The visualized puncture needle therapy is worthy of popularization and further investigation.

## 5. Conclusion

The efficacy of the visualized puncture needle for primary frozen shoulder was better compared to the small needle-knife therapy as discussed in this study. The advantages such as being safer, more convenient, less painful, and more effective were significant. In other words, the visualized puncture needle for primary frozen shoulder is more appropriate and valuable for clinical popularization.

## Figures and Tables

**Table 1:** Comparison of overall efficacy.

Group	N	Cured	Improved	Uncured	Response rate (%)
PN	34	21 (61.76)	9 (26.47)	4 (11.77	30 (88.23)^*★*^
SN	34	11 (32.35)	12 (35.29)	11 (32.36)	23 (67.64)

*Note.* “★”: compared with the control group, *P* < 0.05. PN: puncture needle group; SN: small needle-knife therapy group. All tables are as above

**Table 2:** Comparison of the shoulder scores (mean ± SD).

Group	N	Before treatment	After treatment
PN	34	13.61 ± 3.77	31.22 ± 3.34^*★▲*^
SN	34	14.34 ± 3.89	25.43 ± 3.83^*▲*^

Note: “★”: compared with the small needle-knife group, *P* < 0.05. “▲”: compared with the situation before treatment, *P* < 0.05.

**Table 3:** Comparison of shoulder mobility (°, mean ± SD).

	Group	N	Before treatment	1 week later	2 weeks later	3 weeks later
Abduction	PN	34	84.51 ± 12.79	112.14 ± 9.68^*★*^	118.11 ± 10.81^*★*^	135.13 ± 16.56^*★▲*^
	SN	34	86.17 ± 12.54	93.34 ± 10.44	98.57 ± 11.04	109.34 ± 17.45^*★*^

Forward flexion	PN	34	98.65 ± 16.76	120.51 ± 14.63	134.47 ± 15.77^*★*^	144.32 ± 18.73^*★▲*^
	SN	34	99.12 ± 16.67	108.23 ± 14.55	117.62 ± 13.97	130.32 ± 16.47^*★*^

Backward extension	PN	34	36.37 ± 8.59	38.57 ± 7.87	43.44 ± 8.09	48.87 ± 8.31^*★*^
	SN	34	38.85 ± 9.05	39.57 ± 8.01	40.36 ± 8.55	45.15 ± 10.02

Note: “★”: compared with the situation before treatment, *P* < 0.05. “▲”: compared with the control group, *P* < 0.05.

**Table 4:** Measurement of VAS pain scores (mean ± SD).

Group	N	Before treatment	1 week later	2 weeks later	3 weeks later
PN	34	7.12 ± 1.44	5.31 ± 1.76^*★*^	4.34 ± 1.71^*★▲*^	3.41 ± 1.39^*★▲*^
SN	34	7.21 ± 1.45	6.76 ± 1.56	5.78 ± 1.85^*★*^	5.02 ± 1.76^*★*^

Note: “★”: compared with the situation before treatment, *P* < 0.05. “▲”: compared with the control group, *P* < 0.05.

**Table 5:** Comparison of muscle thickness measured by ultrasound elastography (mm, mean ± SD).

	Group	N	Before treatment	1 week later	2 weeks later	3 weeks later
Supraspinatus muscle	PN	34	12.54 ± 0.76	13.51 ± 0.71	14.26 ± 0.74^*★*^	15.45 ± 0.69^*★*^
	SN	34	12.58 ± 0..68	12.99 ± 0.69	13.58 ± 0.72	13.76 ± 0.63
Infraspinatus muscle	PN	34	16.37 ± 0.59	16.97 ± 0.60	17.37 ± 0.65	18.87 ± 0.66^*★*^
	SN	34	16.85 ± 0.61	16.84 ± 0.65	16.95 ± 0.68	17.05 ± 0.62

Note: “★”: compared with the situation before treatment, *P* < 0.05. “▲”: compared with the control group, *P* < 0.05.

**Table 6:** Comparison of muscle elasticity *E* measured by ultrasound elastography (mean ± SD).

	Group	N	Before treatment	1 week later	2 weeks later	3 weeks later
Supraspinatus muscle	PN	34	3.54 ± 0.37	3.11 ± 0.41	2.96 ± 0.34^*★*^	2.63 ± 0.39^*★▲*^
	SN	34	3.48 ± 0.38	3.21 ± 0.39	3.11 ± 0.42	3.05 ± 0.38
Infraspinatus muscle	PN	34	3.22 ± 0.34	2.97 ± 0.30	2.67 ± 0.35	2.31 ± 0.31^*★▲*^
	SN	34	3.25 ± 0.32	2.94 ± 0.35	2.85 ± 0.38	2.71 ± 0.34

Note: “★”: compared with the situation before treatment, *P* < 0.05. “▲”: compared with the control group, *P* < 0.05.

## Data Availability

The simulation experiment data used to support the findings of this study are available from the corresponding author upon reasonable request.
